The article "Research on the Impact Evaluation of Digital Finance on the Synergy between Economic Development and Ecological Environment" was published in 2022. Journal: J Environ Public Health.

# Research on the Impact Evaluation of Digital Finance on the Synergy between Economic Development and Ecological Environment

**DOI:** 10.1155/2022/1714609

**Published:** 2022-06-29

**Authors:** Feng Yuan

**Affiliations:** School of Economics and Management, JiLin Engineering Normal University, Changchun 130052, China

## Abstract

Following rapid growth, China's economy is entering a period of high-quality economic growth. High-quality economic development has a profound impact on China's current economic development. It can be said that the improvement of economic quality is an inevitable choice for China's new stage of economic development. From this point of view, promoting high-quality economic development has become an important practical issue in my country's current economic and social development. As the integration and innovation of digital technology and taxation, the blessing of digital technology maximizes integration and precision, which can effectively meet the needs of higher stages of economic development. Perfect and inclusive development has become an important support for sustainable and healthy economic development. At present, behind the rapid economic growth, human economic activities have led to the emergence of an ecological and environmental crisis. The growth mode characterized by high input, high consumption support, and high emissions has resulted in insufficient supply of regional ecological and environmental resources, pollution, and damage to the ecological environment and also intensified. Therefore, this paper first examines the concept of digital finance and its enlightenment to economic development, and believes that digital finance has a good role in promoting economic development. Second, an evaluation model for the relationship between environmental environment and economic development is established, and an evaluation index system is obtained. Finally, through the comprehensive evaluation and analysis of economic development and ecological environment, it is concluded that in the era of digital finance, the level of regional economic development has been greatly improved, and my country's regional economic development has been greatly improved, which is significantly faster than my country's ecological environment improvement level.

## 1. Introduction

This note highlights some of the latest developments in this rapidly changing field, and given the nascent and rapidly evolving stages of financial services for smallholder farmers, it is too early to draw firm conclusions from the examples to date. This suggests that the success of mobile-enabled financial services may largely depend on a number of factors [1]. In the past few decades, the financial services industry has developed with the development of digitalization, which is characterized by the improved connectivity and speed of data processing in customer interface and back-office process. Recently, the focus of digitalization has shifted from improving the performance of traditional tasks to bringing new business opportunities and models to financial service providers [2]. Currently, some of the issues related to digital finance are areas that have not been critically addressed in the literature, and if addressed, digital finance can better serve individuals, businesses, and governments [3]. After the financial crisis ended from 2007 to 2010, the financial services industry began to accelerate its transformation. The new business model based on the development of converged technology challenges the current situation of the old traditional industries. It is necessary to review the latest developments in financial services and discuss how these developments affect the financing channels of enterprises and individuals [4]. Today, global finance is the paragon of digital life, a system of knowledge, institutions, and practices whose existence depends on the seamless flow of binary data that intertwine investors, analysts, and trading venues around the world, and digital technology and the various forms of action that take place through digital technologies clearly define contemporary finance [5]. As one of the key areas of domestic scientific development, the government pays special attention to the creation and development of digital technology such as the ability to process large amounts of data, which can accelerate economic growth and maintain national security, including financial security [6]. Through empirical methods and measurements, we find that the impact of human capital on China's economic growth can be achieved indirectly by investing in physical capital, which is different from the performance of OECD countries, a finding that has some implications for China's future regional growth inequality [7]. We analyse the role of law in the economy and assess whether China's formal legal system contributes to stable and predictable expectations of property and contractual rights, a prerequisite for economic growth. The relationship between law and economic development is bidirectional and is a co-evolutionary process [8]. As important regional policies and mechanisms, prefecture-level cities are playing an increasingly important role in China's economic development. Based on Chen Ri's theory of economic development, this paper defines China's economic development from the national and regional levels [9]. After the reform and opening up, our country has developed rapidly. The traditional economic growth model of investment, high consumption, and high emission has led to the increasingly prominent contradiction between China's economic growth and the environment. Empirical studies have shown that the relationship between major pollutant emissions and per capita national income in China does not follow the typical EKC [10]. Based on the economic quality and development growth theory, this paper provides a framework for describing economic development in detail, including physical capital, natural capital, and intellectual capital. The results show that since the reform and opening up, all forms of capital growth have been faster than economic growth [11]. Everyone in the world is completely dependent on Earth's ecosystems and the services they provide, human changes in these ecosystems over the past 50 years have been faster and more extensive than at any time in human history, and many ecosystem services are now degraded, due to actions taken to increase the supply of other services, such as food [12]. Research on fragmented ecosystems has focused on the biogeographical consequences of the formation of habitat “islands” of varying sizes, with little practical value to managers. Therefore, management and research on fragmented ecosystems should focus on understanding and controlling these external influences, and there is an urgent need to develop an integrated landscape management approach that places protected areas in the context of the overall landscape [13]. Data on ecosystem goods and services usually appear on incompatible analytical scales, and a standardized reference framework for comprehensive assessment of ecosystem performance is needed for comparative eco-economic analysis. The second part provides an inventory and matrix that integrate these ecosystem services with key ecological, sociocultural, and economic assessment methods [14]. We review evidence for institutional change related to the resilience of complex adaptive ecosystems in terrestrial and aquatic environments, and the functional role of biodiversity in this context. Evidence suggests that the ability of an ecosystem to produce ecosystem services can suddenly shift from an ideal to a less-than-ideal state [15].

## 2. About the Concept of Digital Finance and Its Impact on Economic Development

### 2.1. Digital Finance

Digital finance is the product of combining traditional financial services with digital technologies such as next-generation Internet technology, Internet of Things, artificial intelligence, big data, cloud services, blockchain, biometrics, and cryptography. Digital finance, Internet finance, and financial technology belong to the same economic family tree. Innovation, reach, and accuracy are core characteristics of digital finance. In recent years, digital technology has entered a period of rapid development, which has also made inclusive financial services an important role in the international community. At the same time, it has solved the problem of digital economic development: “financing is expensive and financing is difficult” in the real economy. The latest practice and application of the principle of financial accelerator is the leading mechanism of economic growth in the era of financial constraints.

According to this definition, the demand for financial services is divided into different levels (Figure 1), and digital finance can be seen as a process of continuously satisfying the demand for financial services. From basic financial services such as savings guarantee and electronic payment, to more complex financial services such as bank credit, investment, and purchasing insurance, the more satisfied you are with financial services, the higher the level of inclusive development will be. Therefore, the definition and measurement of digital finance should not be limited to the process of meeting basic financial service needs, but should also take into account that each target group uses a completely different level of financial services.

### 2.2. Theory of Economic Development

The economic development theory takes developing countries as the research object and examines the development process of the national economy and social structure from economic growth to modernization. Compared with economic growth, economic development has more dimensions, and the economic interests of a country or region are not affected by a single source. Therefore, it can be said that economic development theory is the development and deepening of economic growth theory, emphasizing the continuity of economic activities and the balance and coordination of social development.

### 2.3. The Relationship between Digital Finance and High-Quality Economic Development

Rapid economic development is inseparable from the digital transformation of the financial system. This paper explores the connection between the two, especially to determine the specific impact path of digital development on high-quality economic development. However, the current research is still in the stage of measuring the one-way advancement of digital finance. There are three reasons for this. First, the development of digital finance is inseparable from its economic core. Digital taxation is a new form of financial innovation that combines digital technology with traditional finance. Integrating it into new business formats can promote high-quality economic development. Second, due to the digital nature of digital taxation, digital taxation has special power-law characteristics in the digital age. Finally, compared with traditional taxation, digital taxation expands the scope of services, improves service efficiency, and has a greater impact on high-quality economic growth; that is, digital taxation can accelerate the awareness of high-quality economic growth.

### 2.4. Inclusive Growth

Inclusive growth is a very broad concept, which is of great significance to us, which are developing rapidly. Inclusive growth has two key elements: one is the scientific and rational development of the economy, and the other is the participation of the whole society and the sharing of achievements. Inclusive growth not only pays attention to the speed of economic development but also pays attention to the sustainability of development; that is, it requires not only quantitative growth but also the coordinated development of economy, society, resources, and environment.  Figure 2 examines the mechanism of my country's digital economic development from the perspective of inclusive economic growth by constructing a flowchart, illustrating that the impact of digital economic development on inclusive economic growth varies from region to region, social and ecological mutual inclusion.

## 3. Evaluation Model of the Coupling Relationship between Ecological Environment and Economic Development

### 3.1. Standardization of Evaluation Indicators

There are units in the original evaluation index data, so the dimensions of different indicators are different and cannot be directly compared. According to the influence of different indicators on the relationship between the two, the indicators are divided into positive indicators and negative indicators, and then, the dimensionless processing is as follows:

(1) $$\begin{array}{c} x_{ij}^{\prime }=\frac{x_{ij}-\min\left(x_{ij}\right)}{\max\left(x_{ij}\right)-\min\left(x_{ij}\right)}, \end{array}$$

(2) $$\begin{array}{c} x_{ij}^{\prime }=\frac{\max\left(x_{ij}\right)-x_{ij}}{\max\left(x_{ij}\right)-\min\left(x_{ij}\right)}. \end{array}$$

In the formula, max(*x*_*ij*_) is the maximum value of the indicator and min(*x*_*ij*_) is the minimum value of the indicator.

### 3.2. Determine the Weight of Evaluation Indicators

The concept of entropy originated from heat in physics, and later social sciences used “information entropy” to measure the unknown. If the distribution of the original data of the index is large, it means that the amount of data is large, the index value is small, and the weight is large. On the contrary, the weight corresponding to the index is small. The indicators provided by the entropy method have high reliability. The specific calculation method is as follows: suppose you calculate the weight of the *n* indicators in a certain year of the country.

First, we determine the original matrix *X*=(*x*_*ij*_)_min_ and convert the original indicators into dimensionless standard values according to formulas (1) and (2). The standardized *x*_*ij*_′ is normalized, and the specific formula is as follows:

(3) $$\begin{array}{c} p_{ij}=\frac{y_{ij}}{\sum_{i=1}^{m}y_{ij}}. \end{array}$$

Then, the entropy value and redundancy of each index are calculated so that the original index weight can be determined. Among them, entropy can be expressed as follows:

(4) $$\begin{array}{c} p_{ij}=\frac{y_{ij}}{\sum_{i=1}^{m}y_{ij}}. \end{array}$$

Redundancy is as follows:

(5) $$\begin{array}{c} e_{ij}=\frac{1}{\ln\;m}\sum_{j=1}^{n}p_{ij}\ln\frac{1}{p_{ij}}. \end{array}$$

Indicator weight calculation is as follows:

(6) $$\begin{array}{c} \lambda_{j}=\frac{\eta_{j}}{\sum_{j=1}^{n}\eta_{j}}. \end{array}$$

### 3.3. Comprehensive Index Evaluation Model

We measure the efficiency of each subsystem to measure the ecological environment and economic development, and formulate a comprehensive evaluation model

(7) $$\begin{array}{c} U_{q}=\sum_{j=1}^{p}\lambda_{j}x_{j}. \end{array}$$

Since this study includes two subsystems of the development system, we take (q = 1, 2), since *x*_*j*_ is the general value of the j-th initial index, and *λ*_*j*_ is the weight of the j-th index corresponding to the subsystem. Therefore, this study subtly divides the ecological environment and economic development into four grades according to the current evaluation standards: excellent, good, average, and poor, see Table 1 for more information.

### 3.4. Coupling Model and Criterion

The term coupling comes from physics, which describes the phenomenon in which two (or more) systems or modes of motion influence each other through different interactions, that is, the coordination and promotion of dynamic coupling. It is further subdivided into benign coupling and poor coupling, where benign coupling refers to benign interactions between systems or elements within a system that can be well coordinated, otherwise poor coupling. Therefore, the relationship between ecological environment and economic development can reflect the degree of interaction and influence of the two systems in addition to the factors that affect the economic development and ecosystems of various regions.

This paper refers to the concept of physical weight and coupling and the theory of capacitive coupling coefficient, and expands it into a model for calculating the degree of multisystem interaction. The coupling coefficient is a concept in physics. In the circuit, it is expressed as the tightness of the coupling between components, which is the ratio of the actual mutual inductance (absolute value) between the two inductive components to its maximum limit value. The formula is as follows:

(8) $$\begin{array}{c} C={\left\{\frac{\left(U_{1}\cdot U_{2}\right)\cdots U_{m}}{\prod \left(U_{i}+U_{j}\right)}\right\}}^{\left(1/m\right)}. \end{array}$$

Here, *U*_*i*_ is the value of the extended evaluation index for each subsystem (*i* = 1, 2, 3,  ... , m). Since the model is relatively abstract, it is still necessary to determine that the ecological environment system and economic laws include two subsystems.

In order to clarify the degree of connection, a connection formula for the degree of ecological and economic connection is proposed, as shown in the following formula:

(9) $$\begin{array}{c} C=\left\{\frac{\left(U_{1}\cdot U_{2}\right)}{{\left[\left(U_{1}+U_{2}/2\right)\right]}^{2}}\right\}\;\left(K\geq 2\right). \end{array}$$

In the formula, A has a fitting factor, *k* = 2 in the study, and C is the coupling factor. At the same time, a coordination model of ecological environment and economic development will be introduced, which aims to reflect the connection and coordinated development level of the environmental environment system and the entire economic development system more objectively and truly. It is calculated as follows:

(10) $$\begin{array}{c} D={\left(C\times T\right)}^{2},\\ T=\alpha U_{1}+\beta U_{2}. \end{array}$$

In formula (10), D is the degree of linkage coordination, C is the degree of linkage, *T* is an evaluation index reflecting the overall impact of the two systems on development, and *α*, *β* is an undefined factor. Both the economy and the environment are important to development.

### 3.5. Model Establishment

This research mainly uses three models to study the environmental pollution index and economic growth index. The equations corresponding to the three econometric models are as follows:

(11) $$\begin{array}{c} E_{i}=\alpha +\beta_{1}Y+\varepsilon . \end{array}$$

(12) $$\begin{array}{c} E_{i}=\alpha +\beta_{1}Y+\beta_{2}Y^{2}+\varepsilon , \end{array}$$

In the above formula, *E*_*i*_ is each environmental pollution index (*i* = 1, 2, 3), Y is GDP per capita and is the correlation coefficient; *α* is the model parameter; *β*_1_, *β*_2_, *β*_3_ is the term of random error; equation (11) shows that economic growth and environmental pollution have a simple positive and negative linear relationship, and economic growth leads to the quality of the environment.

#### 3.5.1. Power Function

Both the regional economy and the ecological environment system are a system composed of complex and multifaceted elements. If the contribution of each element of the system to the system development is taken as the goal of system development, the connection and coordination can be developed, and the regional economy and ecological environment can be developed. Development must be viewed as a multifunctional issue. Therefore, according to the decision-making method of the multi-objective system, N objectives can be set for the system, in which the higher the *N*_1_ objective is, the better, the lower the *N*_2_ objective is, and the remaining *N* − *N*_1_ − *N*_2_ objectives are not small and close to a certain value. The function describing the relationship between *M*_*i*_ and *G*_*i*_(*X*) is called a power function and is expressed as the following equation:

(13) $$\begin{array}{c} M_{i}=g_{i}\left[G_{i}\left(X\right)\left(i=1,2,\ldots ,N\right)\right]. \end{array}$$

The total power function can be used to describe the overall operation of the system, and its formula is as follows:

(14) $$\begin{array}{c} K=K\left(M_{1},M_{2},\ldots ,M_{M}\right). \end{array}$$

The higher the value of *K*, the better the coordination of the system, and *α*_*ij*_ and *β*_*ij*_ are the upper and lower bounds of the ordered parameters of the critical point of system stability. Then, the order parameters of each order parameter will have an impact on other links. It is expressed in the following format, that is, the higher the index value, the more positive contribution it makes to the system.

(15) $$\begin{array}{c} \left\{\begin{array}{c} 1,x_{ij}\geq \alpha_{ij},\\ M\left(m_{ij}\right)=\frac{x_{ij}-\beta_{ij}}{\alpha_{ij}-\beta_{ij}},\\ 0,x_{ij}\leq \beta_{ij} \end{array}\right.\;\beta_{ij}<x_{ij}<\alpha_{ij}. \end{array}$$

Negative efficiency indicators, that is, the higher the indicator value, the greater the negative impact on the system, include the following:

(16) $$\begin{array}{c} \left\{\begin{array}{c} 1,x_{ij}\leq \beta_{ij}\\ M\left(m_{ij}\right)=\frac{\alpha_{ij}-x_{ij}}{\alpha_{ij}-\beta_{ij}}\\ 0,x_{ij}\geq \alpha_{ij} \end{array}\right.,\beta_{ij}<x_{ij}<\alpha_{ij} \end{array}$$

In formula *M*(*m*_*ij*_), variable *U*_*ij*_ has a systematic efficiency function, *M*(*m*_*ij*_) represents the satisfaction rate of the indicators to achieve each goal, *M*(*m*_*ij*_)=0 is the least satisfied, and *M*(*m*_*ij*_)=1 is the most satisfied, so there is 0 ≤ *M*(*m*_*ij*_) ≤ 1. Using the above formula, for each in the regional economic and environmental interconnection system, the cost is marked as *X*, *Y*, *T*, respectively. The specific expression is shown in the following formulas:

(17) $$\begin{array}{c} X=\sum_{j=1}^{n}w_{1j}M\left(m_{1j}\right), \end{array}$$

(18) $$\begin{array}{c} Y=\sum_{j=1}^{n}w_{2j}M\left(m_{2j}\right), \end{array}$$

(19) $$\begin{array}{c} T=\alpha X+\beta Y. \end{array}$$

Among them, *w*_1*j*_ is the weight in the economic subsystem; *C*_*t*_ is the weight in the ecological subsystem; *α*, *β* is the impact of changes in the economic and environmental subsystems on the overall development; and *T* is the comprehensive coordination index between economic growth and the environment, reflecting economic growth and the environment overall synergies or contributions.

#### 3.5.2. Coupling Coordination Degree Model

The physical capacitive coupling concept and capacitive coupling coefficients are based on the model:

(20) $$\begin{array}{c} C_{n}=\left\{\frac{\left(m_{1},m_{2},\ldots m_{n}\right)}{\prod \left(m_{i}+m_{j}\right)}\right\}. \end{array}$$

Since there are only two subsystems, we can directly get the degree of coordination, which can be expressed as follows:

(21) $$\begin{array}{c} C_{t}=\left\{\frac{X\cdot Y}{\left[{\left(X+Y\right)}^{2}\right]}\right\}. \end{array}$$

It can not only evaluate the coordination degree of two regional economies and different places but also reflect the relative development level of the region. This paper calls the quantitative index the degree of linkage coordination:

(22) $$\begin{array}{c} D_{t}=\sqrt{{\left(XY\right)}^{2}\cdot {\left(\frac{X+Y}{2}\right)}^{2}\cdot T}. \end{array}$$

Among them, *n* is the level factor, generally *n* = 2. The role of the liaison coordinator is to integrate the local economy and ecological environment, coordinate the development level of the atmosphere and the two, and reduce the situation of weak economic and ecological development. However, an abnormal situation has arisen between the two, and the degree of liaison coordination is more suitable for quantifying and comparing the coordinated development of regional economies and the economic links between regions and regions, and has strong operational capabilities.

## 4. Comprehensive Evaluation and Analysis

### 4.1. Evaluation and Analysis of Ecological Environment and Economic Development

This paper analyses the use of the index weight method to calculate the index weight of the evaluation index system, as shown in Table 2; we calculate the China Environment and Economic Development Index according to the calculation method of China's overall evaluation index in Section 3.3, and the results are shown in Table 3 and Figure 3.

Table 2 shows that in the ecosystem subsystem, the forest coverage rate describes the ecological capacity, industrial waste gas emissions, and fertilization intensity, and reflects the pollution of the ecological environment and its contribution to the environment. In the economic development subsystem, the weight of the two indicators in the indicator layer is greater than 0.9, which indicates a high degree of contribution to economic development.

According to the calculation results in Table 2 and the comprehensive evaluation index calculation method described in Section 3.3, the comprehensive evaluation index *U*_1_ of China's ecology and the comprehensive evaluation index *U*_2_ of China's economic development are calculated, as shown in Table 3, and the trend chart is drawn accordingly (see Figure 3).

As can be seen from Figure 3 and Table 3, since 2000, my country's ecological environment has experienced two stages of development: 1: the overall stage of environmental quality (2000–2006): the development of environmental quality in this stage is unstable and changes in other years. The trend is opposite and usually varies widely. 2. Development stage with good ecological environment quality (2007–2012). Since then, the construction of the ecological environment has been guaranteed by the system. In addition, human activities have also had an impact on the ecological environment in recent years. People pay more and more attention to environmental protection, and the government is also dealing with environmental pollution in multiple directions, and the ecological environment will inevitably be improved and developed.

### 4.2. The Impact of Digital Finance on Economic Development

My country has now entered a new stage of normal economic development. The economic growth seems to be slower than ever, but there is still a good growth trend in general. In addition, the impact of digital taxation on China's economic development is also increasing. First, let us analyse the coverage of my country's digital finance.  Table 4 and Figure 4 show the description of my country's digital finance coverage from 2011 to 2018.

The data results in Table 4 and Figure 4 show that during this period, the average, standard deviation, maximum, and minimum coverage rates of my country's digital economy development all showed an upward trend, indicating that my country's digital economy development coverage rate has increased significantly. The number of people covered by digital finance has increased dramatically, and more and more groups are gaining access to financial products and services, contributing to their economic exclusion.

Second, let us analyse the use of digital finance in my country.  Table 5 introduces the use of digital finance in my country from 2011 to 2018. The trend is shown in Figure 5.

It can be seen from Table 5 and Figure 5 that my country's digital finance is developing continuously, showing an overall upward trend. From 2011 to 2018, the standard deviation of the depth of use of digital finance remained basically unchanged, indicating that the frequency of use of digital finance has increased steadily in recent years, but the average and maximum values have increased year by year, which suggests that digital taxes began to trend upward in 2016. The use of digital finance in my country has developed rapidly since Yu'ebao was launched in 2013.

### 4.3. Dynamic Comparison

According to the calculation formula of interconnection coordination degree described in Section 3.4, the regional economic and ecological environment indicators in my country from 1990 to 2012 and their interconnectivity and coordination, as well as interaction types and correlations, were calculated. The stage of harmonious development of my country's regional economy and ecological environment is evaluated, and the types and stages of the relationship between regional economy and ecological environment are determined, and the representative ones are 1990, 2000, and 2012. The results are shown in Tables 6–8.

The above three tables show that from 1990 to 2012, the economy develops harmoniously, and the ecological environment is also significantly improved, especially for the type of connection, as shown in Figure 6, and the number of areas with weaker regional economies became 16-9-2; the number of synchronized areas will be changed to 10-13-16; and the number of ecologically disadvantaged areas will be changed to 3-7-11. As for the link stage, the number of regions for the low-level link stage becomes 28-11-8; the number of regions for the high-level switching stage becomes 1-15-18; and the number of break-in zones becomes 0-3-3.

### 4.4. Phased Comparison

#### 4.4.1. Comparison from 1990 to 2000

From 1990 to 2000, the average level of coordination between local economy and ecological environment in the five provinces and cities was 1.4, and the coordinated development of local economy and ecological environment was relatively weak. But from the analysis of their state, the development level of my country's regional economic system and ecosystem is in a state of constant change, as shown in Figure 7. It can be seen that the development of the regional economic system is directly related to the development of the ecosystem and Y are the comprehensive evaluation values of the regional economic subsystem and the ecological environment subsystem, respectively; C represents the coupling degree, and *D* represents the coupling coordination degree.

#### 4.4.2. Comparison of 2001–2012

From 2001 to 2012, the average score of regional economic ecology in the five provinces and cities was 0.34, which was much higher than other regions' economic development and ecological environment. Specifically, as shown in Figure 8, from 2001 to 2012, there were significant differences in the level of ecosystems and the degree of coordination between regional economies and ecosystems in different regions of the five provinces and cities. The regional economic and ecological environment level of the five provinces and cities improved.

### 4.5. Comprehensive Analysis Conclusion

From 1990 to 2000, the regional economic development level of the five provinces and cities was significantly improved, the adjustment of the regional economy and the ecological environment was significantly improved, and the connection between the economy and the region was strengthened, but the development level of the ecological environment deteriorated. On the whole, the regional economic backward areas have decreased significantly, and the ecologically backward areas have increased significantly. From this, it can be concluded that the level of regional economic development in my country has been significantly improved, and the level of environmental and ecological development has deteriorated. The development of the environment has improved the linkage.

## 5. Conclusions

The interaction between environmental pollution and economic growth is very important for economic development. The rapid depletion of natural resources and the deterioration of ecological environment have become necessary measures to promote the coordinated and sustainable development of regional economy and environment in China, and digital finance has played an important role in promoting it. The research in this field has started abroad, and we are still in the follow-up stage of foreign research. The relationship between economy and ecological environment has been studied qualitatively and quantitatively from different angles, but there are still some shortcomings in the research: (1) the research on the relationship between economy and ecological environment in China is relatively weak and wide, and basically concentrates on the provincial, municipal, or local level. In China, the research on the relationship between economy and ecological environment rarely involves the relationship between economy and ecological environment at provincial and municipal levels; (2) domestic economic research based on relational modelling and coupling theory is still at the dominant static analysis level in economics. In the future, the research on the linkage process between regional economy and ecological environment should evolve from low-level linkage to high-level linkage, so as to better understand the dynamic process of linkage between regional economic development and ecological environment. More long-term comparative analysis of coordinated development of ecological environment and regional economy and coordinated development in China should be carried out in stages in a long period of time.

## Figures and Tables

**Figure 1:** Hierarchy of financial services demand.

**Figure 2:** Mechanism of the role of digital financial development on inclusive economic growth.

**Figure 3:** Trend of comprehensive evaluation index changes.

**Figure 4:** Trends in coverage and breadth of digital financial inclusion.

**Figure 5:** Depth trend of digital finance usage.

**Figure 6:** Coupling types of five provinces and cities in 1990, 2000, and 2012.

**Figure 7:** Coupling and coordinated development of regional economy and ecological environment in five provinces and cities from 1990 to 2000.

**Figure 8:** Coupling and coordinated development of regional economy and ecological environment in 5 provinces and cities from 2001 to 2012.

**Table 1:** Evaluation criteria for ecological environment and economic development status.

Evaluation coefficient	0–0.3	0.3–0.55	0.55–0.8	0.8–1
Evaluation criterion	Difference	Same as	Good	Excellent

**Table 2:** Weights of evaluation indicators of China's ecological environment and economic development.

Subsystem	Evaluating indicator	Indicator weight
Ecological condition	Land area covered with trees	0.13
	Per capita green area	0.16
	Per capita water resources	0.05
	Industrial wastewater discharge volume	0.09
	Natural population growth rate	0.04

Economic development	Gross domestic product	0.15
	Local fiscal revenue	0.11
	Educational appropriations	0.04
	GDP rate of rise	0.28
	Rural per capita net income	0.13

**Table 3:** Comprehensive evaluation index.

A particular year	Ecological condition	Economic development
2000	0.528	0.014
2001	0.495	0.057
2002	0.458	0.111
2003	0.423	0.171
2004	0.412	0.184
2005	0.395	0.241
2006	0.341	0.311
2007	0.348	0.387
2008	0.396	0.396
2009	0.448	0.472
2010	0.494	0.549
2011	0.416	0.638
2012	0.511	0.713

**Table 4:** The coverage of digital finance development from 2011 to 2018.

Class	2011	2022	2013	2014	2015	2016	2017	2018
Mean	49.08	85.32	114.7	147.5	165.5	177.2	198.7	218.1
Standard deviation	23.81	24.58	24.23	24.07	25.28	26.37	25.49	25.01
Least value	1.86	34.96	66.02	101.6	117.5	131.6	153.8	176
Crest value	99.86	158.6	189.1	220	242.9	254.1	273	290.3

**Table 5:** Depth of use of digital finance development from 2011 to 2018.

Class	2011	2022	2013	2014	2015	2016	2017	2018
Mean	55.33	96.24	131.4	124.4	145.5	195.9	242.8	233.2
Standard deviation	16.59	20.93	25.32	22.6	22.27	17.47	21.45	25.19
Least value	4.29	4.12	61.06	71.06	92.72	160.2	197.3	168.2
Crest value	93.61	170.6	215.3	196.7	223.3	251.4	325.7	316.6

**Table 6:** Coupling types and coupling stages in 1990.

Region	X	Y	C	D	Coupling type	Coordination degree	Coupling stage
Beijing	0.53	0.59	0.28	0.25	Synchronized model	Low coordination	Low-level coupling
Tianjin	0.38	0.42	0.2	0.25	Synchronized model	Low coordination	Low-level coupling
Shanghai	0.59	0.36	0.22	0.23	Environmental lag type	Low coordination	Low-level coupling
Hunan	0.34	0.47	0.2	0.24	Synchronized model	Low coordination	Low-level coupling
Sichuan	0.46	0.38	0.21	0.25	Synchronized model	Low coordination	Low-level coupling

**Table 7:** Coupling types and coupling stages in 2000.

Region	X	Y	C	D	Coupling type	Coordination degree	Coupling stage
Beijing	0.47	0.38	0.37	0.32	Synchronized model	Coordinating	High-level coupling
Tianjin	0.35	0.38	0.38	0.3	Synchronized model	Coordinating	High-level coupling
Shanghai	0.57	0.27	0.51	0.3	Environmental lag type	Low coordination	Run-in stage
Hunan	0.33	0.33	0.35	0.29	Synchronized model	Coordinating	High-level coupling
Sichuan	0.34	0.28	0.37	0.28	Synchronized model	Low coordination	Run-in stage

**Table 8:** Coupling types and coupling stages in 2012.

Region	X	Y	C	D	Coupling type	Coordination degree	Coupling stage
Beijing	0.53	0.33	0.38	0.32	Environmental lag type	In coordination	High-level coupling
Tianjin	0.46	0.33	0.41	0.32	Environmental lag type	In coordination	High-level coupling
Shanghai	0.52	0.24	0.47	0.29	Environmental lag type	Low coordination	High-level coupling
Hunan	0.41	0.37	0.41	0.32	Synchronized model	In coordination	High-level coupling
Sichuan	0.44	0.33	0.46	0.31	Environmental lag type	In coordination	High-level coupling

## Data Availability

The experimental data used to support the findings of this study are available from the corresponding author upon request.
